This article has been retracted.

# Identification of Key Genes and Immune Infiltrate in Nonalcoholic Steatohepatitis: A Bioinformatic Analysis

**DOI:** 10.1155/2021/7561645

**Published:** 2021-09-11

**Authors:** Zhen-yu Jiang, Yi Zhou, Lu Zhou, Shao-wei Li, Bang-mao Wang

**Affiliations:** ^1^Department of Graduate School of Tianjin Medical University, Tianjin, China; ^2^Department of Gastroenterology, General Hospital of Tianjin Medical University, Tianjin, China; ^3^Department of Gastroenterology, The Second Affiliated Hospital of Baotou Medical College, Inner Mongolia University of Science and Technology, Baotou, China; ^4^Key Laboratory of Minimally Invasive Techniques & Rapid Rehabilitation of Digestive System Tumor of Zhejiang Province, Taizhou Hospital of Zhejiang Province Affiliated to Wenzhou Medical University, Linhai, Zhejiang Province, China; ^5^Department of Gastroenterology, Taizhou Hospital of Zhejiang Province Affiliated to Wenzhou Medical University, Linhai, Zhejiang Province, China; ^6^Institute of Digestive Disease, Taizhou Hospital of Zhejiang Province Affiliated to Wenzhou Medical University, Linhai, Zhejiang Province, China

## Abstract

**Background:**

Nonalcoholic steatohepatitis (NASH) can progress to cirrhosis and hepatic carcinoma and is closely associated with changes in the neurological environment. The discovery of new biomarkers would aid in the treatment of NASH.

**Methods:**

Data GSE89632 were downloaded from the Gene Expression Omnibus (GEO) database, and *R* package “limma” was used to identify differentially expressed genes (DEGs) for NASH vs. normal tissues. The STRING database was used to construct a protein-protein interaction (PPI) network, and the Cytoscape software program (Version 3.80) was used to visualize the PPI network and identify key genes. The immune infiltration of NASH was determined using the *R* package “CIBERSORT”.

**Results:**

We screened 41 DEGs. GO and KEGG enrichment analyses of the DEGs revealed the enrichment of pathways related to NAFLD steatosis and inflammation. A PPI network analysis was also performed on the DEGs, and seven genes (MYC, CXCL8, FOS, SOCS1, SOCS3, IL6, and PTGS2) were identified as hub genes. An immune infiltration assessment revealed that macrophages M2, memory resting CD4+ T cells, and *γΔ* T cells play important roles in the immune microenvironment of NASH, which may be mediated by the seven identified hub genes.

## 1. Introduction

Nonalcoholic fatty liver disease (NAFLD) is characterized by hepatic steatosis or the accumulation of triglycerides in hepatic cells [1] and is directly related to obesity, hypertension, insulin resistance, and increased levels of blood lipids [2]. The prevalence of NAFLD has been increasing in recent years as the world economy grows and lives improve, with a global prevalence of about 25%.

NAFLD can progress to a more severe form called nonalcoholic steatohepatitis (NASH). NASH is a serious consequence of the development of NAFLD and is characterized by the abnormal accumulation of liver fat and immune cell infiltration caused by chronic hepatitis and inflammation [3]. Most NASH appears to have the consequence of further developing into liver fibrosis and can lead to serious diseases, such as cirrhosis and hepatocellular carcinoma, some of which are also associated with an increased risk of cardiovascular disease. These factors significantly add to the clinical complexity of such patients and increase the difficulty of clinical management. Even more problematic is the fact that there is currently no effective treatment for NASH-related hepatocellular carcinoma (HCC) [4]. However, the factors influencing the progression from NAFLD to NASH and even to HCC are unclear; although, multiple hypotheses have been proposed, including lipotoxicity, oxidative stress, and proinflammatory mediators [5].

In studies of animal models, it has been found that animals with high fat and cholesterol levels exhibit typical pathological features of NAFLD, including hepato- and splenomegaly, early NASH histopathology, hypercholesterolaemia, elevated serum liver enzyme levels, and increased levels of proinflammatory cytokines [6]. A recent study has shown that fat intake is strongly associated with cognitive decline and increased risk of dementia [7]. Given that the high-fat, high-cholesterol diet associated with NASH has the ability to alter the neural environment and thus cause decline of cognition, studying the mechanisms of NASH is urgent for finding potential therapeutic targets and developing new treatments. However, it is important to elucidate the mechanisms underlying NAFLD in detail, as the prevalence and progression mechanisms of NAFLD are still unclear [8].

Bioinformatics has been widely used as a new approach to explore different disease mechanisms. For instance, it can be used for the early diagnosis and prognostic assessment of cancer by screening tumor-related biomarkers from large data repositories [9]. The method is equally useful for identifying key genes associated with NAFLD and NASH, thus furthering the exploration of the mechanisms underlying the development of NASH [10]. The development of NASH can lead to intestinal malnutrition and brain communication disorders through the disruption of metabolic processes and neurotransmission. A bioinformatic analysis of NASH development will allow us to further investigate the impact of the hepatic-intestinal-brain axis on the development of NASH to develop prevention and treatment strategies.

Therefore, we screened for genes with significantly different expressions in NASH patients and healthy individuals using data obtained from public databases. We then identified key genes, analyzed their potential biological functions, and studied the immune infiltration of NASH to further explore the factors associated with NASH and HCC in the future.

## 2. Materials and Methods

### 2.1. Expression Profile Data Acquisition of NASH

Initially, we chose to search for NASH-associated gene expression datasets in the Gene Expression Omnibus (GEO) database (http://www.ncbi.nlm.nih.gov/).To meet research needs, we set the following standards: (1) data must include normal and NAHS livers, and (2) the samples were from humans. Ultimately, we selected GSE89632 for our study. GSE89632 was based on the GPL14951 platform Illumina HumanHT-12 WG-DASL V4.0 R2 expression beadchip. The dataset of GSE89632 includes 63 valid samples, including 20 with simple steatosis (SS), 19 with NASH and 24 health controls (HCs).

### 2.2. Data Process and DEGs of NASH Identified

We downloaded the gene expression matrix of GSE89632 and the annotation file of GPL14951. First, we replace the ID of the probe with the gene symbol, and if they have the same probe, the max one will be retained. According to the aim of our study, we retained expression profiling data for only 24 HCs and 19 NASH patients. As the data had already been processed in a “quantile normalized” fashion, we proceeded directly to the next analysis. The “limma” package was used to identify differentially expressed genes (DEGs) between NASH patients and HCs; genes were considered DEGs if they had |logFC | >2 and *P* value <0.05.

### 2.3. GO and KEGG Enrichment Analyses

GO and KEGG enrichment analyses were used to explore the potential biological functions of DEGs in NASH patients and HCs. The package “clusterprofiler” was used to implement the analysis procedure described above, and the analysis results were presented as bubble plots via the package “ggplot2.”

### 2.4. Protein-Protein Interaction (PPI) Network and Hub Gene Identified

The PPI network of DEGs was constructed by the String dataset (https://www.string-db.org/). The minimum required interaction score was set to 0.4, and the disconnected nodes in the network were hidden. We exported the result obtained by the String database in “TSV” format and subsequently imported it into the Cytoscape software program (Version 3.80). The function “MCODE” of Cytoscape was used to explore the key module, and “cytohubba” was used to identify the hub genes from the network. Default settings were adopted for both “cytohubba” and “MCODE.”

### 2.5. The Assessment of Immune Infiltration in NASH

CIBERSORT, a tool for evaluating the proportions of 22 subtypes of human immune cells, was used to evaluate the immune infiltration of NASH. We chose to calculate the immune infiltration using the “*R*” software program, among the perm was set at 1000. Results were visualized by multiple graphics. Boxplots were used to demonstrate the overall immune cell infiltration in NASH, and a stacked histogram was used to visualize infiltration in individual samples. A *t*-test was used to determine the different infiltration between NASH patients and HCs, and the results were depicted by boxplots. We constructed a correlation matrix of the seven hub genes and TME of NASH, and package “corrplot” was used for visualization.

## 3. Results

### 3.1. Identification of DEGs in NASH

To guarantee the accuracy of the DEGs, we set a *P* value <0.05 and [log2foldchange (log2FC)] > 2 as the cut-off criteria. Ultimately, 41 DEGs were identified, most of which (33/41; 80.49%) were downregulated in NASH patients, with only a small proportion (8/41; 19.51%) upregulated. Volcano plots were used to depict DEGs, with green indicating downregulated genes, red upregulated genes, and gray genes with unsatisfactory conditions (Figure 1(a)). The heat map illustrates the expression profiles of the 41 DEGs in the 2 groups, with blue representing the NASH group, green the HCs, red the DEGs with upregulated expression, and dark blue the DEGs with the downregulated expression (Figure 1(b)).

### 3.2. Results of the Function Enrichment Analysis of 41 DEGs

The occurrence of diseases often involves a variety of biological functions. We therefore used the 41 DEGs to describe significant pathways that might be involved in NASH. A GO enrichment analysis revealed the pathways of “female pregnancy,” “multi−multicellular organism process,” “cellular response to extracellular stimulus,” “response to lipopolysaccharide,” “cellular response to external stimulus,” “response to molecule of bacterial origin,” “response to glucocorticoid,” “response to corticosteroid,” “fat cell differentiation,” and “response to organophosphorus” to be involved in the process of NASH (Figure 2(a)). Furthermore, the KEGG enrichment analysis suggested that the pathways of “osteoclast differentiation,” “IL−17 signaling,” “TNF signaling,” “Janus kinase/signal transducer and activator of transcription (JAK/STAT) signaling,” “microRNAs in cancer,” “prolactin signaling,” “growth hormone synthesis,” “secretion and action,” “type II diabetes mellitus,” “leishmaniasis,” and “colorectal cancer” might be biological pathways altered in NASH compared with normal tissues (Figure 2(b)).

### 3.3. Identification of the DEG PPI Network and Hub Genes

We set the minimum required interaction score at 0.4 when performing the PPI network analysis of DEGs using a string database, hiding the connected nodes in the network. This network totaled 39 nodes with 69 edges, and the vast majority of the constituent networks were downregulated genes. We visualized the network using the Cytoscape software program. As shown in Figure 3(a), blue represents downregulated genes, while red represents upregulated genes. We subsequently analyzed the module via the MCODE function and finally obtained two key modules (Figures 3(b) and 3(c)). The larger module scored 6.571, including “NR4A1,” “MYC,” “CXCL8,” “FOS,” “SOCS3,” “IL6,” “PTGS2,” and “SOCS1.” The other module included “FOSB,” “JUNB,” and “FOSL1,” scoring 3. Goth core modules included downregulated genes, demonstrating the importance of downregulation and the interaction of these genes in NASH. To identify the key candidate genes from the network, we analyzed the main network using cytohubba and obtained the top 10 genes (see Table 1), of which 7 were included in the larger submodule; we identified these 7 genes as hub genes.

### 3.4. Immune Cell Infiltration in NASH and Its Relationship with Hub Genes

The 22 human immune cell proportions of NASH are shown in Figure 4(a). The top three categories were M2 macrophages, T cell CD4 memory resting, and *γΔ*T cells. These three categories accounted for a large proportion of NASH immune cell infiltration (>50%).  Figure 4(b) shows the proportion of immune cell subtypes in individual samples, and it can be seen that there are differences in the infiltration of each sample, but macrophages and T cells comprised a larger proportion of each sample than other subtypes.  Figure 4(c) shows the different immune cell occupancies in NASH and normal liver tissue. M2 macrophages, T cell CD4 memory resting, and *γΔ*T cells were significantly increased in NASH patients compared with HCs, which is again consistent with the high percentage of these cells in NASH patients, underscoring the importance of these three cell types in the immune microenvironment of NASH.

Subsequently, we explored the relationship between the seven hub genes and the tumor microenvironment (TME) in NASH. “Naïve B cells,” “plasma cells,” “*γΔ*T cells,” “monocytes,” “M2 macrophages,” “resting mast cells,” and “activated mast cells” showed a consistent correlation among the seven hub genes, indicating that these genes are involved in the formation of the specific immune cell infiltration pattern of NASH.

## 4. Discussion

NASH is characterized by the abnormal accumulation of liver fat and immune cell infiltration due to chronic inflammation, which can lead to liver diseases, such as cirrhosis and hepatocellular carcinoma, and is strongly associated with cognitive decline and an increased risk of dementia in response to an altered neuroenvironment. The discovery of new biomarkers is therefore important for identifying potential therapeutic targets and developing new treatments.

To investigate the underlying biological mechanisms contributing to the development and progression of NASH, we performed GO and KEGG analyses of DEGs and identified many significant biological pathway enrichments. Th17 cells and IL-17 have been proven to promote the transformation from simple steatosis to steatohepatitis, which is closely related to NAFLD steatosis and inflammation [11]. The JAK-STAT signaling pathway has also been proven to be involved in the regulation of NASH. Abnormalities in the GH-JAK2-STAT5 signaling pathway altered the whole-body fat metabolism to promote peripheral lipolysis while enhancing hepatic fat synthesis, resulting in hepatic fat accumulation and leading to the development of the NAFLD phenotype [12].

We also performed a PPI network analysis of DEGs and identified seven hub genes: “MYC,” “CXCL8,” “FOS,” “SOCS1,” “SOCS3,” “IL6,” and “PTGS2.” MYC is a protooncogene encoding a nuclear-phosphorylated protein that plays a role in cell cycle progression, apoptosis, and cell transformation. Amplification of the MYC gene has been observed in a variety of cancers. In liver disease, highly aggressive and poorly differentiated HCC has been shown to be significantly associated with its overexpression [13]. Activation of the MYC gene has also been observed in HCC cells in mouse experiments [14]. After knockout of the MYC gene, the livers of mice developed NAFLD-specific and progressively similar features to NASH [15]. In our study, MYC was also found to be downregulated in NASH patients, which is consistent with the above studies and further suggests that MYC may be an important factor affecting hepatic lipid metabolism.

Chemokines are chemoattractants for leukocyte trafficking, growth, and activation in injured and inflammatory tissues. As inflammation is key in the transition from SS to NASH, chemokines may play an important role in the pathogenesis of NASH. There is growing evidence that the expression of chemokines and their receptors is elevated in the livers of obese patients with advanced steatosis and NASH [16]. CXCL8 is a member of the CXC chemokine subfamily secreted by these cells, which primarily regulates the recruitment of neutrophils to sites of inflammation. It has been shown that serum CXCL8 levels are significantly higher in patients with NASH than in those with SS or HCs. Meanwhile, CXCL8 is an essential multifunctional cytokine that promotes tumor metastasis and invasion [17]. It has been confirmed that HCC patients with an increased expression of CXCL8 always had a worse outcome than those with a low expression [18]. CXCL8 was mapped to the pathways related to LPS, TRL3, B cells, monocytes, and the KEGG toll-like receptor signaling pathway. However, the specific role of CXCL8 in the pathogenesis of NASH remains unclear, meriting a further indepth study [19].

The fos gene, or c-fos, is a major member of the fos gene family, which regulates transcription from promoters containing AP-1 activation elements. C-fos acts as a natural partner of c-jun to promote cell growth. However, the overexpression of c-jun protein in the absence of c-fos may lead to the abnormal formation of homodimer transcriptional complexes, thus disrupting the normal regulation mechanism of gene expression [20]. In studies of liver disease, c-jun has been shown to be strongly expressed in the liver of patients with acute hepatitis. In a NASH mouse model, c-Jun/AP-1 activation was found to be a key regulator of liver changes. An increase in c-jun may promote the development and progression of NASH [21]. Since the DNA binding domain of c-fos is homologous to the c-Jun DNA binding domain, we may speculate that c-fos also plays an important role in the occurrence and development of NASH [20]. In the occurrence and development of HCC, the liver-specific c-fos expression leads to reversible premalignant hepatocyte transformation and enhanced dEn-carcinogenesis. c-fos-expressing livers show necrotic foci, immune cell infiltration, and an altered hepatocyte morphology. Furthermore, increased proliferation, dedifferentiation, activation of the DNA damage response, and gene signatures of aggressive HCCs are also observed. Mechanistically, c-fos decreases the expression and activity of the nuclear receptor LXr*α*, leading to increased hepatic cholesterol and the accumulation of toxic oxysterols and bile acids [22]. Therefore, the role of c-fos in the disease progression of NASH or HCC is contradictory and mysterious, meriting further research [23].

Cytokine signaling repressor proteins (SOCS1-SOCS7 and cytokine-induced SH-2 containing proteins) are induced by proinflammatory cytokines and regulate cytokine signaling through the JAK/STAT pathway [24]. SOCS1 and SOCS3, as suppressors of cytokine signaling, have both been found to be associated with insulin resistance. However, the role of SOCS3 is more paradoxical and deserves to be explored [25, 26]. In NASH, the increased inflammatory response leads to an increase in inflammatory factors, such as interleukin-6 (IL-6)3 and tumor necrosis factor-*α* (TNF-*α*), which in turn leads to an increase in the SOCS3 expression [27]. SOCS3 protein is thought to promote insulin resistance by inhibiting insulin and leptin signaling in the inflammatory response. However, in mice, hepatic SOCS3 deficiency was found to enhance hepatic insulin sensitivity but paradoxically promotes NAFLD and inflammation in a hypertrophic environment with high glucose and fatty acids [28]. These findings reveal that SOCS3 plays an important negative regulatory role in insulin sensitivity, adipogenesis, and energy homeostasis as well as having a complex role in promoting the development of NASH. At the same time, SOCS3 is known to inhibit cytokine signaling via JAK/signal transducers, activators of transcription, NF-*κ*B, and the focal adhesion kinase (FAK) signaling pathway. Substantial data have demonstrated the link between the SOCS3 regulation of inflammation and its suppressor activity on tumor initiation and development. In SOCS3 conditional knockout mice, deletion of the SOCS3 gene promoted carcinogen-induced hepatic tumor development through the activation of STAT3 and resistance to apoptosis. In HCC patient samples, the expression of SOCS3 was reduced compared with surrounding non-HCC regions [29]. Recently, hypermethylation of SOCS3 was shown to be associated with a poor clinical outcome in HCC patients with hepatitis B virus (HBV) infection backgrounds but not in those with hepatitis C virus (HCV) or no virus infection [30].

IL-6 is an inflammatory factor produced primarily at sites of acute and chronic inflammation. The IL-6 expression is significantly higher in steatotic livers than in normal livers, suggesting that IL-6 is involved in the progression of NASH [31]. It has also been found that IL-6 levels correlate significantly with NASH severity [32]. However, our results do not seem to support the above, as we found the IL-6 expression to be downregulated in NASH. The role of IL-6 in liver injury is complex and contradictory. IL-6 has been found to promote hepatocyte regeneration [33], impede apoptosis, and repair damaged cells [34] after liver injury. This suggests that the role of IL-6 in liver cells is multidirectional and not merely proinflammatory, which is well worth further study.

Prostaglandin-endoperoxide synthase (PTGS), also known as cyclooxygenase, is a key enzyme in prostaglandin biosynthesis. There are two isozymes of PTGS: constitutive PTGS1 and inducible PTGS2, which together are involved in prostaglandin biosynthesis during inflammation and mitosis. PTGS2, or cyclooxygenase-2, was found to be significantly associated with iron death, a new type of cell death that has been recently reported and extensively studied. Iron death is characterized by the contribution of iron to the development of oxidative cellular damage. Current studies suggest that it may be associated with different types of chronic liver diseases, including HCV, NASH, and HCC, as well as DILI. An imbalance in iron metabolism and reactive oxygen species- (ROS-) induced lipid peroxidation is thought to be mechanisms involved in the liver injury sustained in these diseases [29, 35, 36]. Furthermore, PTGS2 has been identified as a marker of iron sagging, along with other markers, including changes in NADPH levels and lipid peroxidation [37, 38]. However, the effect of PTGS2 on NASH has yet to be investigated.

NASH has a chronic inflammatory manifestation and has been shown to have multiple immune cells directly associated with it. We analyzed the immune infiltration in the liver of NASH patients compared to normal patients using CIBERSORT and found significant differences in multiple subtypes of immune cells between HCs and NASH patients. The correlation between the seven hub genes and immune cells also revealed consistency in the expression of these genes with multiple immune cells. For example, all seven hub genes were underexpressed in NASH patients compared with HCs (Figure 3), and the expression of these genes was positively correlated with naïve B cells (Figure 4(d)), while the proportion of naïve B cells was reduced in NASH patients compared with HCs (Figure 4(c)). Taken together, we conclude that the low expression of these hub genes may mediate the decline in multiple immune cells associated with NASH. Those genes may be involved in shaping the immune microenvironment characteristic of NASH, but the exact mechanisms remain to be investigated.

The immune infiltration analysis showed that the proportion of M2 macrophages, memory resting CD4+ T cells, and *γΔ* T cells was significantly elevated in NASH compared with normal hepatic cells, indicating the importance of these three types of immune cells in the immune microenvironment of NASH. The pathology of NASH is characterized by lipid-induced hepatocyte apoptosis and inflammatory cell infiltration, some of which are activated macrophages [39]. Macrophages have a unique phenotype and function. They are generally considered to be involved in the inflammatory response to NASH [40, 41]. Excessive lipid accumulation in the liver promotes the activation of Kupffer cells (KCs) and the production of inflammatory mediators (TNF-*α* and IL-1*β*, among others), leading to increased insulin resistance, liver inflammation, and the formation of the blood-brain barrier, which eventually results in the development of NASH [42]. M1 macrophages have the capacity to deliver antigens and secrete proinflammatory cytokines, whereas M2 macrophages downregulate the immune response by secreting the inhibitory cytokines IL-10, transforming growth factor-*β* (TGF-*β*,) and mannose receptor (Mrc) [43, 44]. Dysregulation of M1/M2 macrophages can lead to chronic inflammation, cancer, and NAFLD [45]. In recent years, it has been suggested that M2 macrophages may play a protective role against NAFLD by promoting apoptosis of M1 macrophages. However, the observation in our study that M2-like cells are much more abundant than normal cells in NASH seems to contradict the above view. This may be explained by the plasticity and flexibility of mononuclear phagocytes and their activation state, i.e., that polarized M1/M2 macrophages can reverse the phenotype to some extent both in vivo and in vitro [45, 46]. Another view is that the increase in M2-like cells is a consequence rather than a cause of NASH. The progression of NAFL to NASH is accompanied by apoptosis and repair of hepatocytes, and the increase in M2 macrophages may thus be related to hepatocyte repair and chronic inflammation of the liver.

As NASH is a chronic inflammatory disease, hepatic CD4+ T cell infiltration becomes a feature of NASH. An increase in human CD4+ central and effector memory T cells in the liver and peripheral blood has been observed, accompanied by a significant upregulation of proinflammatory cytokines (IL-17A and interferon gamma). Furthermore, the clearance of CD4+ T cells was shown to reduce liver inflammation and fibrosis in mice, and a study by Rau et al. highlighted an increase in CD4+ memory T cells at sites of intrahepatic fibrosis in patients with NAFLD, demonstrating that CD4+ memory T cell subsets are important drivers of progression from steatosis to fibrosis in NAFLD. However, there is a lack of directly relevant studies and explanations for the role of memory resting CD4+ T cells in NASH. Our findings may serve as a hint for future directions.

*γΔ* T cells belong to a unique subset of innate lymphocytes. They can produce at least two distinct subsets: interferon- (IFN-) *γ*- and interleukin- (IL-) 17-producing *γΔ* T cells. *γΔ* T cells play a protective role in several pathophysiological processes, such as pathogen clearance, tumor surveillance, and tissue repair, while playing the opposite role in autoimmunity, allergy and carcinogenesis [47]. Thus, the role of *γΔ* T cells in maintaining immune homeostasis and tissue homeostasis is complex and bidirectional, with these cells acting as both “protectors” and “destroyers.” There is growing evidence that *γΔ* T cells in the liver respond to liver-targeted injury and regulate the development of liver disease [48, 49], thus playing an important role in maintaining liver physiological homeostasis as well as regulating liver pathological processes. NAFLD is a chronic progression of the liver from SS to cirrhosis, while NASH is an important pathological change in the middle of this progression [50]. It has been shown that IL-17 accelerates the progression of NAFLD by recruiting neutrophils and inducing ROS [51]. *γΔ* T cells are the main supplier of IL-17A [52]. An increase in IL-17A-producing *γΔ* T cells can be seen in mice with NAFLD. *γΔ* T cell deficiency protects mice from NAFLD damage, characterized by steatohepatitis IL-17A in CD161+ *γΔ* T cells [48]. Thus, IL-17A-producing *γΔ* T cells are a major regulator of the progression of NAFLD. However, there is still a lack of corresponding studies on the mechanisms underlying the direct and indirect effects of *γΔ* T-cell subsets on NASH. The mechanism underlying the activation of *γΔ* T-cell subsets also remains a mystery. Our findings of an increased and active expression of *γΔ* T cells in NASH patients corroborate previous findings and may highlight a potential therapeutic approach to blocking the progression of SS to NASH and eventually to NAFLD, via blocking or eliminating IL-17A-producing *γΔ* T cells.

## 5. Conclusion

We identified seven hub genes that are closely related to the development of NASH through a bioinformatics analysis and also clarified the immune infiltration of NASH through an immune cell subtype analysis, providing a useful reference for future research on NASH biomarkers and the immune microenvironment.

## Figures and Tables

**Figure 1:** Differentially expressed genes (DEGs) in NASH vs. normal tissues. (a) A volcano plot of all DEGs. (b) Heat map of DGEs.

**Figure 2:** A functional enrichment analysis of DEGs shown by bubble plots. (a) The results of a GO enrichment analysis. (b) The results of a KEGG enrichment analysis.

**Figure 3:** A functional protein-protein interaction (PPI) network. (a) PPI network of DEGs of NASH. Blue represents downregulated genes, while red represents upregulated genes. (b, c) Key modules of the PPI network.

**Figure 4:** Immune infiltration in NASH. (a, b) The proportion of 22 immune cell subtypes in NASH. (c) The 22 subtypes of immune cells have different proportions in NASH and normal tissues. (d) Correlation matrix: blank represents no correlation, red represents a positive correlation, and blue represents a negative correlation.

**Table 1:** Top 10 DEGs in the network ranked by the MCC method.

Rank	Name	Score
1	IL6	1101
2	FOS	1082
3	MYC	926
4	CXCL8	774
5	PTGS2	769
6	SOCS3	744
7	SOCS1	726
8	FOSB	294
9	FOSL1	264
9	JUNB	264

## Data Availability

The data used to support the findings of this study are included within the article.
